The article "“Doing a good thing for myself”: a qualitative study of young adults’ strategies for reducing takeaway food consumption" was published in 2019. Journal: BMC Public Health.

# “Doing a good thing for myself”: a qualitative study of young adults’ strategies for reducing takeaway food consumption

**DOI:** 10.1186/s12889-019-6731-3

**Published:** 2019-05-07

**Authors:** Anne C. Grunseit, Amelia S. Cook, Janet Conti, Melissa Gwizd, Margaret Allman-Farinelli

**Affiliations:** 1 Sydney School of Public Health, University of Sydney Prevention Research Collaboration, Sydney, Australia; 2 School of Science and Health, Western Sydney University, Sydney, Australia; 3 School of Social Sciences and Psychology, Western Sydney University, Sydney, Australia; 4 Charles Perkins Centre, University of Sydney School of Life and Environmental Sciences, Sydney, Australia

**Keywords:** Qualitative, Young adults, Fast foods, Take-away foods, Behaviour change, Ready-to-eat meals

## Abstract

**Background:**

Increasingly the population is eating meals and snacks prepared outside the home, especially younger adults. Takeaway foods can be energy-dense, high in saturated fat and sodium, and deleterious to health. Extending studies examining the barriers to healthy eating, this paper explores strategies employed by young adults who report reducing consumption of unhealthy takeaway foods.

**Methods:**

Young adults aged 18 to 35 years in paid employment were recruited to participate in eight semi-structured focus groups. In response to initial findings, recruitment for the final four groups refocused on participants who either wanted, were in the process of, or had changed their takeaway food habits. Focus group recordings were transcribed verbatim and coded by two researchers for recurrent themes using an inductive method.

**Results:**

Forty-eight participants with a mean BMI of 23.4 kg/m^2^ and mean age of 25 years took part, of which 34 were female, and 27 were born outside Australia. Four broad strategies emerged: altering cognitions about consumption/reduction of takeaway food; practical changes to behaviours; finding external support; and, reconfiguring social events. In detail, participants cognitively recast takeaway food consumption as negative (expensive and unhealthy) and reducing consumption of such foods or consuming healthy alternatives as a (positive) self-care action. Setting goals and making personal rules around consumption, and consciously making practical changes, such as planning for food shopping, were other strategies. Externally derived support including supportive food environments and friends and family passively reduced exposure to unhealthy takeaway food. Finally, some participants actively created social environments supportive of healthy choices.

**Conclusions:**

Our participants reported strategies they believed led to them successfully reduce their takeaway food consumption by matching the attractions (e.g., convenience) and countering apparent disincentives for reducing consumption (e.g., losing a reward) of takeaway food. They reported eschewing more short-term rewards and costs, to prioritise their health, believing that avoiding these foods would benefit them personally and financially. The identified strategies are consistent with documented techniques for successful behaviour change and corresponded to all levels in the social-ecological model from intrapersonal factors to public policy. The findings could underpin health promotion strategies to support this at-risk group.

## Background

Overconsumption of takeaway foods (TAF) has been a cause for concern for public health practitioners as they are often high in energy, total fat, saturated fat, and sodium [1]. Although what is considered to comprise this group of foods varies between studies, it is typically broader than fast food and could include cold and hot foods purchased for immediate consumption from fast food and casual restaurants, cafeterias, and snack bars. It may also include foods taken away, or delivered, from full table service restaurants and cafes (i.e. eaten elsewhere). Therefore, one broad definition of TAF has been ‘any meal prepared outside the home that, when bought, is ready-to-eat as a meal’ [2]. A recent review reported links between TAF and increased obesity, fast food and increased daily energy intake, out-of-home eating and increased saturated fat and total fat intake [3]. Despite the associated health risks, TAF constitutes a significant proportion of the diet in countries such as the US, UK and Australia [3]. For example, it has been estimated that in the UK one third of the daily energy comes from food prepared outside the home [4] and at last assessment, 36% of Australian adults consumed food prepared outside the home in a 24-h period [5]. Further, meals out and fast foods accounted for over 34% of Australian on ‘Food and non-alcoholic beverage’ household spending [6].

Young adults represent a particularly at-risk group in terms of TAF consumption and its short and long-term health sequelae. Firstly, this group are among the highest consumers of TAF in the UK, Australia and the US [7–9] and accordingly spend more on fast food and TAF than any other age group. For example, as a proportion of ‘Food and non-alcoholic beverages’ and ‘Total goods and services expenditure’ Australian 15–24 year olds spend 19.4 and 3.0%, and 25–34 year olds spend 16.5 and 2.7%, respectively compared with 13.1 and 2.2% for all households [6]. Secondly, a prospective study of young adults aged 18–30 years in the US found that compared with infrequent consumers of fast food, those consuming fast food more than twice per week gained 4.5 kg more weight over 15 years [9]. Australian research also shows the 20–30 years age bracket is a period of acceleration in obesity rates [10] and young adulthood is associated with a generally poorer diet with low fruit and vegetable intake [11] and high consumption of sugar-sweetened beverages [12]. The most frequent consumers of TAF among young Australian adults according to one survey tend to be male, younger and single [13]. Finally, food behaviours seem to track over time and a lack of involvement in food preparation during early adulthood is associated with poorer diet quality during the mid- to late-twenties [14].

Previous research shows that changing food habits long-term towards a healthier pattern may be difficult. For example, Australian research indicated that a variety of factors support continuation of energy-dense beverage consumption such as feeling part of a social group, competitive pricing versus non-energy dense options and the health consequences of consumption being considered remote and not personally relevant [15]. Other research showed similar themes, but also noted how negative constructions of healthy food amongst adolescents as without taste and healthy eating as an unpleasant, short-term activity further shored up the attractiveness of energy-dense foods. Little formative research, however, has been conducted on how young Australians can change [16] and how health promotion programs may be better designed to support this behaviour. By contrast with previous research addressing barriers [15, 16], here we describe strategies and other factors reported by young adults who believe themselves to have been successful in decreasing their consumption of TAF in order to elucidate how they have overcome such barriers.

## Methods

### Participants

Participants were recruited from March 2011 to May 2012 from one Australian university and its surrounds using on-campus posters and advertisements in staff and student e-newsletters. A recent meta-analysis has shown that more than 60% of university/college students gain weight during the first year of attendance, with a mean gain of 3.38 kg (95% confidence interval, 2.85–3.92) [17] showing they are a group at particular risk. Convenience and snowball sampling was used to recruit current or recent regular TAF consumers who met the eligibility criteria of being aged 18 to 35 years with a source of income, from working or a scholarship stipend, to enable food purchases independent of parents. This recruitment strategy inadvertedly initially attracted healthy eaters with a keen interest in good nutrition, therefore, partway through the study, the recruitment materials and eligibility criteria were modified to attract people who were consumers of TAF. They needed to (1) be wanting to change; (2) be in the process of changing; or, (3) have recently changed, their TAF eating habits. In addition, due to the disproportionate numbers of females in the initial focus groups, some recruitment materials advertised specifically for males to ensure the findings were more representative of the population. The study was approved by The Institutional Human Ethics Research Committee (approval number: 13497). Informed, written consent was obtained from all participants.

### Procedure

Semi-structured discussions were facilitated by two interviewers who were present in each focus group (ASC and JC). A discussion guide was developed by the interviewers using a motivational interviewing framework [18] with the intention of generating participant narratives which tapped into participants’ motivation to change in addition to what might hinder change talk. More specifically, questions were generated which gathered respondents’ accounts of their current TAF consumption habits, interest in and motivations for changing TAF consumption and their experience of trying to reduce TAF consumption where it had been attempted. Questions included: attractions, detractions and concerns of TAF; frequency, types, and situations of TAF consumption; personal concern/acceptability of own consumption and situations where it may increase/decrease; acceptable frequency of TAF consumption; and, experiences of decreasing TAF consumption. Focus groups were conducted until no new themes emerged (thematic saturation). Each group was audiorecorded using a digital recorder and later transcribed in conversational style with speaker identification.

Following the focus group interview, participants completed a socio-demographic questionnaire and self-reported their height and weight. Body Mass Index (BMI; kg/m^2^) was calculated and participants were categorised into underweight (< 18.5 kg/m^2^), normal weight (18.5–24.9 kg/m^2^), overweight (25.0–29.9 kg/m^2^) or obese (≥30.0 kg/m^2^). Distribution of socioeconomic status was determined using the postal area-based Socio-Economic Indexes for Areas using the Index of Relative Socio-economic Advantage and Disadvantage [19]. These data were collected for descriptive purposes such that the sample here may be compared with other research.

### Qualitative analysis

The qualitative data underwent iterative thematic analysis with a view to producing a framework and content for an intervention to reduce TAF consumption amongst young adults. Themes relevant to this aim were generated from the content of the interviews, grounded in the understandings and lived experience of a sample of this group, rather than formulated a priori consistent with an inductive approach. A coding frame was developed (AG) and discussed and modified in collaboration with two other researchers (ASC and MG). We then coded the data following a thematic inductive approach as described by Braun and Clarke [20]. Themes relevant to understanding what participants thought constituted TAF, factors affecting their purchase and consumption of TAF, and triggers and strategies for maintenance of reduced intake of TAF were generated. To ensure consistent coding, one transcript was coded independently by AG and MG and the coding compared. Discrepancies were discussed and further modifications were made to the coding frame. The remainder of the transcripts were divided and coded separately by (AG and MG). In the second stage, data were retrieved and reanalysed for recurrent themes through an iterative process whereby commonalities in explanations were identified along with exceptions and tested against the data (AG). The data were analysed using QSR NVivo version 10.0.

## Results

### Sociodemographic and anthropometric characteristics

Nine focus groups were conducted, ranging in size from three to eight participants (a total of 51 participants). The average length of each focus group was 67 min. One group (Group 5, *n* = 3) was excluded from analysis because two participants were nutrition researchers and the third participant was a research exercise physiologist as it is likely their perceptions and attitudes towards TAF would differ substantially from those of the non-expert population for whom an intervention would be developed. Of the eight groups that were analysed, two were female only (Group 4, *n* = 6; Group 7, *n* = 4) and one group was male only (Group 9, n = 3). Of the remaining 48 participants, 34 were female (71%), 27 were born outside Australia (56%), and the mean age was 25.3 years (sd = 4.9). A high proportion had a university degree (62.5%). One in five participants were overweight or obese and the mean BMI was 23.4 kg/m^2^ (sd = 4.4). Twenty-two were employed in full time work (≥ 35 h per week) and 26 in part-time work or on a scholarship stipend.

### Takeaway foods - definition

Although we asked participants for their own definitions of what constituted the concept of “takeaway foods” at the beginning of the discussion, following this discussion the researchers made clear the foods that were to be considered for the remainder of the discussion concerning reducing TAF consumption. These foods were described as: high fat TAF that are prepared outside the home and bought ready-to-eat. For example, fast food like cheeseburgers, hamburgers, pizzas, fries and other foods that may be commonly purchased outside the home and eaten outside the home, like meat pies, sausage rolls, roast or fried chicken or fried fish along with other takeout meal options such as Chinese, Thai, and Indian TAF.

### Reducing takeaway food consumption

Not all participants in the focus groups had tried to reduce their TAF intake, and a number had tried to do so but not been successful. Therefore, whilst the analysis included the whole dataset (excluding Group 5 as noted above) the data reported in detail here comprises the strategies and factors which participants described which they believe assisted them to achieve a reduction in TAF consumption if and when it happened. We have adopted this approach instead of a more conventional one of identifying barriers to reduction, as it can serve to demonstrate the means by which young people themselves address the barriers they encounter [21] and serve to underpin intervention development.

### Strategies to reduce consumption of takeaway foods

The discussion with young people who felt they had successfully reduced their intake of TAF could be summarised into four main themes: 1) Recasting consumption and/or reduction of TAF; 2) Practical changes to behavioural practices shaping food choices; 3) External instrumental support; and, 4) Reconfiguring social events and TAF. We have ordered of the themes in terms of those which contributed most to understanding the data are discussed first, followed by more minor themes [22].

Each of the themes is reported below, with illustrative quotes from the discussion groups in Table 1. It should be noted that these main and sub-themes were by no means mutually exclusive and participants certainly reported using more than one strategy. However, for the purpose of the paper, we will first detail the content of these strategies, their similarities and differences, and then note how they intersected with each other and/or clustered according to characteristics of the participants.

**Table 1:** Illustrative quotes of themes and sub-themes from young adults

Theme	Sub-theme	Illustrative quote
1. Recasting consumption and/or reduction of TAF	1.1 Self-care action	… but I hit a tipping point with going, I am not being managed properly; and then I just started to do that. So I was pushed to an extreme, I guess, before I was like, right, now it’s time to prioritise. K, Group 2, 32yo female, full-time employed, lives with peers
		…having that I don’t have to be around my friends all the time, for every moment. I don’t mind missing things now and taking more care of myself becomes more important, basically, because you get older and you see how your body changes and things. J, Group 2, 22yo female, full-time employed, lives with partner & peers
		Maybe if every time you make that decision, you should say you’re doing it not because you hate your fat body; it’s because you love your body and you love your health. You’re not making a decision out of resenting the way you are or the way that you might perceive yourself, but that decision you make at that point in time is like, I’m doing myself a favour here…I’m doing a good thing for myself. SS, Group 8, 33yo female, full-time employed, lives alone
	1.2 Reaching a goal	I guess, if I’ve got a goal and - it’s a bad way of thinking but it’s just my frame of mind, would be if there’s something that I need to achieve or need to lose weight for, I’ll possibly do it, but then other times, I don’t really think about it. OO, Group 7, 30yo female, full-time employed, lives with partner & children
		Well, I got married in December, so it was like before that, both me and my wife kind of were not eating it [TAF] every week, but we were eating it fairly regularly, and trying to just be healthier and be a bit slimmer, and also save a bit more money to the wedding. LL, Group 6, 32yo male, full-time employed, lives with partner
	1.3 Saving money	I guess it can be kind of cost-effective as well. Like my loaf of bread can last a week, and I try and eat the mandarin if I get hungry and stuff, so I guess that makes me feel good to not eat other things. HH, Group 6, 23yo female, full-time employed, lives with partner & children
		…last year, I was eating [takeaway foods] several times a week, and consistently every Friday night with all my family, we’d have takeaway. But now I’m working Friday nights and I’m working more and trying to save up money and everything, so I’ve been reducing the amount I eat out… U, Group 3, 19yo male, part-time employed, lives with parents
	1.4 Small changes	… I don’t want to think about food, I don’t want to have discussions about food, I don’t want to discuss with anyone eating, I just made sure I exercised and let myself eat bad things once in a while. But not, perhaps, as much as otherwise. So going the extreme is too much, it’s not realistic and that’s what’s slowly helped me just doing it bit by bit. K, Group 2, 32yo female, full-time employed, lives with peers
		Inversely, if you think about the long term as a series of decisions, you can say, okay, if I make the right decision every single time, or say eight out of 10 times, that’s a better way to think about it than, okay, I’m going to change my eating habits long-term. VV, Group 8, 24yo male, part-time employed, lives with parents
2. Practical changes to behavioural practices shaping food choices	2.1 Planning	…when I cook for myself and if it’s over a long period of time, what I do is I make a lot of one thing in one go and then I just stick it in the fridge so I can come back to the same thing. …it just means that I’m not eating out like takeaway foods, but it’s still just in the fridge. P, Group 3, 20yo female, part-time employed, lives with parents
		It just suits my lifestyle. It’s like I’m used to doing it, so I pack food every day. Q, Group 3, 18yo male, part-time employed, lives with parents
	2.2 Rule-making	You’re like, oh well, there’s nothing really in the fridge that I want to take for lunch or - I don’t really have time to go home for dinner so maybe I should just - so then I really try to identify, okay, how often have I done that this week or this month. And say no, that has to be - I have to go home even if there’s nothing in the fridge. AA, Group 4, 23yo female, part-time employed, lives with parents
		So what I have implemented is do all my shopping on Saturdays and stay back at home on Sundays, all social things on Saturdays and just stay back home on Sundays. So Sundays, I’ll cook at home, and no food from outside that day. RR, Group 8, 29yo female, employment status unknown, lives with partner
	2.3 Portion adjustment	…but now we try to have one dish for two. Now we try to adapt and say, okay, we know that last time it was too much, so we try to think before. FF, Group 6, 32yo female, part-time employed, lives with partner & children
		I don’t think that’s fair… I don’t like not being able to reduce the size of the portion I’d like to have quite easily. That would make me feel not as guilty if I ate a smaller amount of it, without having to choose not to eat as much that’s on my plate. UU, Group 8, 34yo female, full-time employed, lives with partner
3. External instrumental support	3.1 Food environment	I also think considering we’re not taking into account all the sushi and salads and whatever, I think that helps as well because you can be in a food court and someone can choose Hungry Jack’s and you can choose a healthy option. MM, Group 7, 23yo female, full-time employed, lives with partner
		Living at the parental home gives you a base of healthy food to draw on, especially if your parents are healthy people, but then that’s decisive. If you’d moved out of home and you don’t have that, you’ve just got a shelf with a few scattered items on it, then it forces your hand to eat takeaway food. S, Group 3, 23yo male, part-time employed, lives with peers
		… when I was in Canada and America when you go to Macdonald’s they have the kilojoule content of each item on the menu next to it, and I found that it did affect my choices. I, Group 2, 32yo female, full-time employed, lives with peers
	3.2 Social support	And so that really helped, because it was both of us deciding together as well. LL, Group 6, 32yo male, full-time employed, lives with partner
		I guess, just the overall goal, and my husband is being very encouraging at the moment, so he’s giving me time to go exercise and he’s chipping in with helping cook. So yeah, it’s just changes together. OO, Group 7, 30yo female, full-time employed, lives with partner & children
		Living at the parental home gives you a base of healthy food to draw on, especially if your parents are healthy people, but then that’s decisive. If you’d moved out of home and you don’t have that, you’ve just got a shelf with a few scattered items on it, then it forces your hand to eat takeaway food. S, Group 3, 23yo male, part-time employed, lives with peers
4. Reconfiguring social events and takeaway foods		It’s a bonding thing. Like we’ll get a movie and we’ll watch - like you’re in the living room in front of the TV instead of in the kitchen. It’s - you can do that with pizza. AB, Group 4, 27yo female, part-time employed, lives with peers & partner
		Or if I met up with friends in a takeaway food setting I would be discreet about it because I wouldn’t want to ruin the atmosphere of celebrating with takeaway food, but I’d be discreetly just participating in the atmosphere, not the food part of it. I, Group 2, 32yo female, full-time employed, lives with peers
		I do enjoy cooking, so when I do put the time to it, and because you’re linking it with a social thing, I don’t feel like I’m wasting time, because then we sit and eat it and have wine, but you know, it’s still healthy. M, Group 3, 19yo female, part-time employed, lives with parents.

#### Recasting consumption and/or reduction of takeaway foods

When participants discussed the attractions of TAF, they were often described through dichotomies positioning TAF in a positive construction and in opposition to homemade foods in a negative construction. These dualisms included: time and effort saving (versus time consuming); a reward for working or studying hard (versus doing more work by shopping and cooking food); and, a symbol of being freed from restrictions of “being good” or “being healthy” (versus with being restrictive and boring).

Through these understandings, TAF held positive valence when contrasted to home-prepared food. Casting TAF in these positive roles seemed to grant participants license to overlook the well-recognised health impact of regularly consuming TAF. When those who reported being successful in reducing the amount of TAF they consumed described the strategies that they used, one group of approaches was to recast TAF consumption as negative; correspondingly avoiding or reducing consumption of these foods or consuming healthy alternatives had a positive value. Four sub-themes characterised the re-conceptualisations of reductions in TAF consumption: a “self-care” action; part of reaching a goal; saving money; and, a series of small changes in habit.

##### Self-care action

A number of participants described how reducing TAF and/or choosing healthier foods was understood as a means by which they took care of themselves and prioritised their health before the attractions of TAF as described above. For example, one participant described how she felt her boss was forcing her into working long hours which in turn meant she was eating a significant amount of TAF and not exercising. Her reduction of such foods was symbolic of her not accepting unreasonable work demands that led to her compromising her health (Table 1, Sub-theme 1.1). Another participant linked this with getting older and the changing of priorities that come with age. In her case, she changed the way she conducted her social life placing a healthier lifestyle before accepting all social invitations which inevitably involved eating fast food (Table 1, Sub-theme 1.1). Others talked about reducing consumption as part of “respecting” themselves or loving their body. Borrowing on a discourse of self-care to structure food choices allowed these participants to recast consumption of TAF as something not in their own self-interest and therefore of negative value.

##### Moving towards a goal

Participants who believed they had successfully reduced their TAF consumption found that working towards a goal helped shift their food habits. Many had weight loss for a particular event or purpose as the galvanising goal (Table 1, Sub-theme 1.2). A helpful cognitive strategy for some participants was having a goal that was not directly about reducing TAF for its own health benefit but rather, in the service of another aim. Weight loss itself was not always an end in itself either but linked to another goal such as wedding or pregnancy which lent further impetus for change. One drawback of this approach, however, was once the goal was reached, the value of avoiding TAF may be lost (Table 1, Sub-theme 1.2).

##### Saving money

Although cost is one of the first mentioned attractions of TAF in this sample, some participants identified the increasing cumulative cost of such foods as an impetus to change food habits (Table 1, Sub-theme 1.3). Young adults are especially price sensitive as they may be at a life stage when earnings are not high, and life events such as moving out of home, marriage, travel and having children place an extra strain on budgets [23, 24]. Recognition of the true financial cost of eating TAF in combination with the goal of saving money provided a positive framing for a reduction of TAF consumption.

##### Small changes

In contrast to having a long term goal, a third sub-theme under cognitive recasting was to focus on the immediate choices to be made about food in the belief that this would make reductions in TAF less overwhelming. Rather than “being extreme”, changes in habits were made by stealth or “bit by bit” as one participant explained (Table 1, Subtheme 1.4). Another participant described his cognitive mechanism of redirecting attention towards the small, immediate decisions which would accumulate to a long-term habit (Table 1, Sub-theme 1.4). Both approaches appear to be seeking to make a potentially large shift in food habit cognitively manageable by focussing on immediate and discrete behavioural choices.

#### Practical changes to behavioural practices shaping food choices

A second major theme in participants’ descriptions of how they believed they achieved a reduction in TAF consumption included those that involved applied and practical strategising. Sub-themes included: planning; rule-making; and, portion adjustment.

##### Planning

Planning is an often recommended strategy in weight loss/maintenance [25] and was a tactic reportedly employed by our participants. Planning might take the form of ensuring sufficient stocks of food at home, cooking ahead (bulk cooking), building a repertoire of quick-to-make recipes, or packing food to take to university or the workplace (Table 1, Subtheme 2.1). Participants reported having a strategy in place that may pre-empt being in a situation where the person is hungry but has something that is time and cost efficient. Such planning neutralises one of the main ‘advantages’ attributed to TAF, that of convenience, by making homemade foods equally convenient at the point where the food choice is being made.

##### Rule-making

Some participants described consciously making a rule around TAF, most commonly, limiting TAF frequency. Other manifestations of rule-making centred on quarantining the times or circumstances in which TAF can or cannot be eaten (Table 1, Subtheme 2.2). Rule-making created a boundary which mitigated against unknowingly consuming excessive TAF; a rule forces the person to audit their intake and measure it against what they had decided apriori was reasonable.

##### Active TAF portion control

A final practical behavioural means used by this sample to reduce TAF intake was through conscious control over portion size. An extended discussion took place in one group (Group 6) with a number of participants describing a range of portion-control strategies such as putting only half of a serve of TAF on the plate and refrigerating the rest or delaying going for a second serve, or buying less (Table 1, Subtheme 2.3). One participant described a counter-intuitive situation where buying the larger serve actually works in favour of portion control because she used satiety cues to stop eating, whereas with a smaller serve, she would eat until the serve was finished. Another group talked about potentially buying children’s meals at a fast food chain because they are smaller, but expressed frustration because this option was not open to customers aged over 12. In this group of strategies, the adjustment of consumption occurs on occasions where TAF is actually bought, so is contained within a TAF consumption event rather than prior to a decision to buy, as the ‘planning’ strategy is. The approach seems to work by foreclosing on excessive intake by buying or serving an amount which makes it impossible or more difficult to eat too much.

#### External instrumental support

The two categories of strategies described above involve a high degree of agency on the part of the person wanting to reduce intake. That is, the individual actively generates, for example, cognitive frames which supported their wish to eat less TAF, or actively implements practical strategies which would counteract some of the attractions of TAF, or aim for a goal which lends a positive valence to a reduction in TAF intake. A third major theme in participants’ description of what assisted them with reducing their consumption of TAF referred to external factors which participants felt aided them to reduce TAF consumption. There were two main sub-themes that we identified: Food environment and social support.

##### Food environment

As described above, some participants who were successful in reducing their TAF consumption created personal food environments which supported them not buying TAF. However, the participants also talked about being in situations where they did not have control over the range of foods they could choose from, for example when they were outside the home and/or with friends. Being able to make choices about foods to eat, even when in an environment that included energy-dense TAF options, was important. Two participants in Group 7 had an exchange on this point which was typical of discussions in other groups (Table 1, Subtheme 3.1). Their quotes refer to healthier options being available across TAF outlets, and within menus of particular outlets. Others referred to cost of energy-dense versus healthier options shaping food choices in such situations. Another mentions menu-labelling influencing her of food choice within the range of TAF (Table 1, Subtheme 3.1). Thus, although participants had strategies that they could enact to minimise choosing TAF, in situations where they were faced with choosing from among food options they had no control over, the range, price and accompanying information was important in maintaining their resolve to limit TAF intake.

##### Social support

A number of participants mentioned that having a supportive partner assisted with cutting down on TAF consumption (Table 1, Subtheme 3.2) and the support given could be in the form of a shared decision or goal, or providing instrumental support with assistance in cooking. While many of the participants gave negative examples where they were undermined by their social connections, a small number described where their efforts to reduce TAF were made easier when those with whom they share meals did not work against them. For young people living at home, the preparation of meals by parents also assisted making the choice to not eat TAF simpler.

Thus the two sub-themes above describe factors which participants felt assisted them in reducing TAF consumption, but unlike themes 1 and 2, were more passive in that these were factors over which they had less personal agency.

#### TAF and social interaction

For this group of young adults, social context was closely bound to TAF consumption. Social events are held at TAF outlets, late nights out finish with a visit to a fast food shop because it is the only food amenity open, or there were enjoyable social rituals with a TAF component (e.g., a Sunday night treat) (Table 1, Theme 4.0). Many discussed the numerous mechanisms at play when social interactions worked against reducing TAF consumption such as peer pressure, not wanting to be the ‘odd one out’, or missing out on a social occasion altogether. For those successful at reducing TAF however, a number of solutions to these challenges were described. For example, one participant actively couples a home prepared meal with a social occasion, where once a week she and a friend cook for each other (Table 1, Theme 4.0). The overarching strategy for those who were successful at reducing TAF, was to uncouple eating TAF from pleasurable social occasions either through gravitation away from groups that had that pattern, or modifying interactions with those groups. For others, the social aspect was linked to home-prepared meals transferring the social dividend to healthier meals. Negotiating the social consequences of not wanting to have TAF was fraught but also possible.

## Discussion

Research has shown that young people report challenges in trying to reduce the amount of TAF they consume [26]. Factors such as perceived lower cost, taste, and convenience are cited as reasons which guide them towards choosing energy-dense TAF and away from healthier homemade options [27–29]. The current study describes a number of strategies that young people, who report reducing their TAF consumption, have found useful in navigating those barriers. These include increasing awareness of their own worth and individual identity as a healthy person; knowledge that TAF does not cost less than healthier foods; setting personally specific, achievable, timely goals; creating opportunities to avoid TAF by planning meals ahead and improving their food environment; and deriving motivation through social support and reconfiguring their social networks to enable improved meal choices. The strategies used address the attractions and justifications for consuming TAF. For example, where TAF is convenient, planning makes a home-cooked meal more convenient; where social interaction involves TAF, a communal cooking effort confers a social dividend; where TAF is a reward, a healthy choice is being good to oneself; where the rate of consumption is invisible, rule-making renders it visible and auditable; and finally, where TAF is seen as time and cost-efficient, cooking home-made food ahead and in bulk yields time and cost savings.

The informal strategies described by the participants resonate with other research including those that have reviewed and/or tested more formal behaviour change approaches to weight loss and/or promotion of healthy eating. For example, corresponding to our rule-making (2.2) and reaching a goal (1.2) sub-themes two systematic reviews have found that interventions that promote self-monitoring and goal setting are effective in achieving healthier eating [30, 31]. In a meta-analysis of randomised controlled trials, these factors were found to be independent predictors of short (≤6 months) and long (≥12 months) term dietary and/or physical activity improvements, although these trials were conducted in overweight and obese adults [30]. In terms of a mechanism, making rules about food consumption fosters self-regulation, a noted enabler for weight management, by setting boundaries around eating behaviour [31]. To follow the rule, one must both self-monitor one’s behaviour for compliance and compare the behaviour to the desired behaviour. With respect to goal-setting, this is most often described in terms wanting to reach a certain weight or some other risk factor or health goal [25]. Of interest here, is that the goals described by our participants were not solely related to eating behaviour but other priorities such as weight loss for a personal purpose like a wedding or pregnancy planning. Therefore, interventions aimed at reducing TAF consumption which is defined in terms of a behaviour (e.g., eat fewer takeaway meals) may perhaps be most effective when linked with other personally relevant but non-health related goals.

Samdal et al. [30] also found the behaviour change techniques of graded tasks and barrier identification/problem solving to be significant predictors of healthy eating in the short term which correspond to our small changes (1.4) and modifying social interaction sub-themes (4.0). Graded tasks break down a target behaviour into short term steps (e.g., buy a healthier option this one time) which people may find easier to adhere to, and in the case of our participants, to imagine themselves performing than a broader long term goal (reduce TAF consumption). Wing et al. (2016) have also shown that small changes in food intake and physical activity can prevent weight gain as shown in a group followed for up to three years [32]. Thus, the strategy suggested by the participants in the current study may prove effective for improving their diet longer term. Problem solving, on the other hand, requires thinking ahead about potential barriers to a long term behaviour goal and generating a solution [25]. As noted by the participants in our study, during adolescence eating TAF becomes a social norm and peer group pressure to eat these foods is strong and this may persist during young adulthood [33]. The participants anticipated being exposed to TAF and put strategies into place that could still bring them social benefits without having to consume unhealthy TAF by either inconspicuously not eating the food or participating in communal cooking. Young people willing to use these strategies could be further assisted through more supportive public food environments (see discussion below).

In agreement with previous survey research, we found that time [28, 34] and cost [23, 35] were two factors drawing participants to TAF. However, with respect to the former while these participants acknowledged the convenience of TAF, they reported planning ahead could counteract the need for it. Australian research has demonstrated that allocating less time to eating can predispose to higher TAF consumption [8]. In focus groups with college students in the US, researchers identified that having time to plan to shop, cook and clean up after meals was a motivator to home food preparation and home cooking could save money [36]. Therefore, time management and availability seem to be key factors to be taken into account when planning interventions for young adults to reduce TAF consumption. Knowledge of the true comparative costs may additionally be considered an enabling factor motivating them to avoid TAF as also postulated by others [37].

Our findings have also resonated with a number of qualitative studies examining healthy eating. For example, the cognitive recasting which these participants described which repositioned not eating TAF as “doing a good thing for myself” (Table 1) is consistent with a qualitative study of 40 adolescents and young adults who had successfully lost weight. [38]. The authors contend that the primary motivation to make changes to diet and physical activity was an internally derived desire for better health and elevated their sense of their own self-worth. Another study used focus groups with adults (mean age 34.2 years) in Ireland to investigate their views on views about what influenced portion size selection and management. Participants reported purposefully buying food (not just TAF) in portion-controlled sizes or portioning and storing appropriate serving sizes was one strategy to assist better portion control [39]. Whilst TAF presents some particular challenges as portion sizes are often excessive [40], our participants exercised very similar approaches by reducing how much they served to themselves and storing the remainder or sharing their takeaway meal. However, the complaint that they were prohibited from buying the inherently smaller “kids portion” speaks to the importance of the wider food supply system and how individual intentions are situated within broader contexts and therefore somewhat constrained in a more or less supportive environment.

When people are hungry they will eat what is available and therefore food environments where consumers have reduced control over selection are extremely important in influencing diet. In the Coronary Artery Risk Development in Young Adults cohort for example, low income respondents’ proximity to fast food restaurants was positively associated with consumption [41], although others have found no relationship between the frequency of fast food consumption and proximity to outlets [42]. Whether recognition prompts intake or internal motivation makes one more observant of food sources is uncertain but the range of foods in physical and temporal space limited the ease with which our participants could minimise TAF consumption. They did, however, recognise both the chains selling more nutritious food and the addition of healthy items to the menus of food chains with menus predominated by high energy, high saturated fat, high sodium foods. Some also said that menu-labelling influenced their choices. A study undertaken at the same University from which the current sample was recruited found that awareness of the labelling after some social marketing was just over 40% but for those who noticed and wanted to use the information (9%) it did result in lower energy food selections [43]. Nikolaou et al. (2014) found calorie-labelling in a university-cafeteria resulted in 3.5 kg less weight gain in students over a one year period [44]. Therefore, whilst food environments vary widely in terms of how much they may challenge an individual’s commitment to reducing TAF, providing healthier menu items and nutritional information at least broadens opportunities if not selected options.

What is salient about the strategies and factors described here is that they traverse the spectrum of the social-ecological model, especially as explicated by Fitzgerald and Spaccarotella (2009) [45]. This model posits that health-related behaviours are affected by factors operating at different levels from the personal characteristics of individuals to the macrosystems of culture and public policy. Our participants referenced intrapersonal strategies on perceptions and knowledge and skills through the cognitive recasting and using the caloric and financial cost of TAF to motivate change. They also referred to strategies which were interpersonal; benefitting (albeit passively) from positive social support but also actively changing food availability where they could and building social relations which supported healthy eating. Moving further outward in the model, they modified portion sizes and engaged with problem solved in food environments external to the home. Finally, their strategies interacted with broader culture as they sought to find ways to still participate but still not consume TAF. Importantly this means that in order to support the types of strategies that young adults might find appropriate, those support strategies need to operate at a range of levels and not merely involve individual education as many programs do [46].

The issue of agency is pertinent here. Whilst on the one hand many of the strategies and techniques described by our participants were highly agentic [46] in that the participants talked about drawing on their own resources to change, those solutions may be augmented and perhaps rendered more powerful if they are surrounded by supportive multilevel action. For example, young people’s desire to take care of their health through healthy eating but have no time to home-prepare food can be assisted by providing mostly healthy food options in places which they frequent such as tertiary education institutions. A desire for convenient, affordable social eating might be supported by facilities that network young people for communal cooking. In other words, high agency actions may be further supported by low agency environmental restructuring which may incrementally increase the probability of a healthy choice. Although some of our participants implied a need for macrolevel change, given the importance of autonomy to this subpopulation with respect to their health [38] and the comparatively lower acceptability of government-led diet interventions restricting or eliminating choice [47] careful consideration would need to be given to framing and implementation.

The insights gained through this analysis provide new and useful information from which interventions may be planned in future to offset the perceived barriers to eating less TAF. The strength of the study is that we have used the reported experiences of young adults themselves to inform solutions. Further, the strategies were from those who report that they have successfully reduced their consumption and therefore reflected mechanisms that had been generated under real-world circumstances. There are however some limitations of the current study. The scope of the findings are limited by the low numbers of males and overweight or obese participants. Hence, the range of strategies to reduce TAF among these groups may not have been fully captured in our focus groups. The students mostly lived in areas of higher socioeconomic status (although they themselves mostly were not earning high incomes) and involved in tertiary education. Therefore, they may have been able to draw on resources which other subpopulations may not and the strategies identified here may not be successfully implemented by young adults from different socioeconomic and educational backgrounds. Initially we recruited participants who were female and eating very healthy diets with minimal intake of TAF and therefore we needed to re-focus the recruitment strategy to gain new insights from consumers. However, it is not unusual for sampling strategies to change in response to preliminary analysis in qualitative research and indeed is important they do so in order to maximise saturation [48]. Finally, this is analysis is formative and any intervention developed from these data would require an evaluation of effectiveness and scalability to population level.

## Conclusion

Young people can and do reduce their consumption of TAF successfully using a range of strategies that address not only the attractions of TAF, but the apparent disincentives for reducing consumption. Interventions directed at the individual level should include goal-setting, self-monitoring, nutrition education to discern between unhealthy and healthy TAF to increase skills and confidence in preparing nutritious meals, as well as tapping into a person’s instrinsic motivation to change. Recommendations for environmental level change include increasing the availability of healthy alternatives, reducing the cost of healthy choices in line with or below the price of unhealthy options, and introducing labelling to help the quick identification of healthy choices. Building a social and wider food environment supportive of the healthy food choices an individual aspires to, may provide a valuable leverage point to work against many of the attractions of TAF.

## Abbreviations

BMI: Body mass index
TAF: Takeaway food
